# Development and Validation of a Risk Prediction Model for Ventricular Arrhythmia in Elderly Patients with Coronary Heart Disease

This article has been retracted.

**DOI:** 10.1155/2021/2283018

**Published:** 2021-07-02

**Authors:** Ying Dong, Yajun Shi, Jinli Wang, Qing Dan, Ling Gao, Chenghui Zhao, Yang Mu, Miao Liu, Chengliang Yin, Rilige Wu, Yuqi Liu, Yang Li, Xueping Wang

**Affiliations:** ^1^Department of Cardiology, First Medical Center of Chinese PLA General Hospital, Beijing, China; ^2^Graduate School of Chinese PLA General Hospital, Beijing, China; ^3^National Engineering Laboratory for Medical Big Data Application Technology, Chinese PLA General Hospital, Beijing, China; ^4^Medical Big Data Research Center, Medical Innovation Research Division of Chinese PLA General Hospital, Beijing, China; ^5^Faculty of Medicine, Macau University of Science and Technology, Macau, China

## Abstract

**Background:**

Sudden cardiac death is a leading cause of death from coronary heart disease (CHD). The risk of sudden cardiac death (SCD) increases with age, and sudden arrhythmic death remains a major cause of mortality in elderly individuals, especially ventricular arrhythmias (VA). We developed a risk prediction model by combining ECG and other clinical noninvasive indexes including biomarkers and echocardiology for VA in elderly patients with CHD.

**Method:**

In the retrospective study, a total of 2231 consecutive elderly patients (≥60 years old) with CHD hospitalized were investigated, and finally 1983 patients were enrolled as the model group. The occurrence of VA within 12 months was mainly collected. Study parameters included clinical characteristics (age, gender, height, weight, BMI, and past medical history), ECG indexes (QTcd, Tp-e/QT, and HRV indexes), biomarker indexes (NT-proBNP, Myo, cTnT, CK-MB, CRP, K^+^, and Ca^2+^), and echocardiology indexes. In the respective study, 406 elderly patients (≥60 years old) with CHD were included as the verification group to verify the model in terms of differentiation and calibration.

**Results:**

In the multiparameter model, seven independent predictors were selected: LVEF, LAV, HLP, QTcd, sex, Tp-e/QT, and age. Increased HLP, Tp-e/QT, QTcd, age, and LAV were risk factors (RR > 1), while female and increased LVEF were protective factors (RR < 1). This model can well predict the occurrence of VA in elderly patients with CHD (for model group, AUC: 0.721, 95% CI: 0.669∼0.772; for verification group, AUC: 0.73, 95% CI: 0.648∼0.818; Hosmer–Lemeshow *χ*^2^ = 13.541, *P*=0.095). After adjusting the predictors, it was found that the combination of clinical indexes and ECG indexes could predict VA more efficiently than using clinical indexes alone.

**Conclusions:**

LVEF, LAV, QTcd, Tp-e/QT, gender, age, and HLP were independent predictors of VA risk in elderly patients with CHD. Among these factors, the echocardiology indexes LVEF and LAV had the greatest influence on the predictive efficiency of the model, followed by ECG indexes, QTcd and Tp-e/QT. After verification, the model had a good degree of differentiation and calibration, which can provide a certain reference for clinical prediction of the VA occurrence in elderly patients with CHD.

## 1. Introduction

Sudden cardiac death is a leading cause of death from coronary heart disease (CHD). Sudden cardiac death affects approximately 3 million people worldwide each year, more than the deaths from breast, lung, and colon-rectum cancers combined [1]. The risk of sudden cardiac death (SCD) increases with age, and sudden arrhythmic death remains a major cause of mortality in elderly individuals [2]. Although SCD can occur due to a slow heart rhythm (bradycardia) caused by stopping or blocking of the normal sinus pacemaker, more commonly, it is due to a rapid heart rhythm (tachycardia), usually originating in the ventricles—ventricular tachycardia (VT) or ventricular fibrillation (VF) [3]. Studies indicate that 50%–85% of sudden cardiac deaths are attributed to ventricular arrhythmias (VA) [4, 5].

Due to myocardial ischemia and partial myocardial tissue necrosis or fibrosis in patients with CHD, abnormal cardiac electrophysiological remodeling occurs, which is easy to induce VA. ECG indexes can reflect the electrophysiological changes of the heart. Although there were some studies that incorporate ECG indexes into the prediction model of clinical events [6–10], there was still a lack of large sample research on the combination of multiple ECG parameters for VA in elderly patients with CHD. Previous researches paid more attention to the relationship of one single ECG index and VA [11, 12], while myocardial electrical activity is actually influenced by multifactors. One single ECG index is far from enough to reflect the myocardial electrical activity.

The aim of this study was, therefore, to develop a risk prediction model by combining ECG and other clinical noninvasive indexes including biomarkers and echocardiology for VA in elderly patients with CHD. We first retrospectively investigated the relationship between various indexes and VA in elderly CHD patients, hoping to establish a model to predict VA. Then, we prospectively collected data to verify the model in terms of differentiation and calibration.

## 2. Methods

### 2.1. Study Population

Originally, a total of 2231 consecutive elderly patients (≥60 years old) with CHD hospitalized at Chinese PLA General Hospital from January 2010 to December 2016 were investigated retrospectively. The occurrence of VA within 12 months was mainly collected. The patients with no complete clinical information were excluded. Finally, 1983 patients who had complete data were enrolled as the model group.

A total of 513 elderly patients (≥60 years old) with CHD who were hospitalized in the same unit from January 2017 to December 2018 were included as the verification group. The results of a 24-hour ambulatory electrocardiogram were collected respectively at the first hospitalization, 6 months, and 12 months after hospitalization. The occurrence of VA events was observed. Finally, 406 patients with complete data were included.

Inclusion criteria for the subjects were as follows: aged over 60 years; clinically diagnosed as CHD. In both the model group and verification groups, we excluded patients with secondary ST-T changes caused by various causes, such as congenital heart disease, valvular heart disease, cor pulmonale, hypertensive heart disease, preexcitation syndrome, intraventricular conduction block, and pacemaker implantation. In addition, patients who have taken amiodarone or long-term chemotherapeutic drugs within one month, which may affect the QT interval and T-wave morphology, were also excluded [13, 14].

All the patients signed informed consent forms, and the study complied with the Declaration of Helsinki and was approved by the Research Ethics Board of our center.

### 2.2. Electrocardiogram Measurement

Electrocardiography used a standard digital recorder (GE, MAC 5500) with 12 simultaneous leads at a paper speed of 25 mm/s.

#### 2.2.1. QTcd

Upon each lead, a smooth and clear baseline for 3 consecutive QT intervals was measured, and the mean value was calculated [15]. In order to eliminate the effect of heart rate on the results, the Bazzett formula was used to correct the QT interval, and the correction value was QTc: $\text{QTc}=\text{QT}/\sqrt{\text{RR}}$. QTc_max_ and the QTc_min_ were selected in the synchronous standard 12-lead ECG, and then QTcd was obtained: QTcd = QTc_max_ − QTc_min_.

#### 2.2.2. Tp-e

Tp-e was measured in three consecutive cardiac cycles, and the mean values were calculated [16]. Tp-e was defined as the interval from the peak of a positive T-wave or the nadir of a negative T-wave to the end of the T-wave. The QT interval of lead V3 was measured and the correction value QTc was calculated. Tp-e and QTc values were input into the computer, and the Tp-e/QTc ratio was calculated. All ECG measurements were performed independently by two physicians blindly. When the measurement results were inconsistent, the average was calculated.

### 2.3. Ventricular Arrhythmias

A 24 h 12-lead dynamic electrocardiograph was used for data acquisition, including heart rate variability (HRV) indexes and VA. The range of VA included [17] cardiac arrhythmia ≥3 consecutive complexes originating in the ventricles at a rate of >100 bpm (cycle length: <600 ms), torsades de pointes, ventricular flutter, and ventricular fibrillation.

## 3. Statistical Analyses

In univariate analysis, the categorical variables were expressed by frequency and percentage, and Pearson's chi-square test or Fisher's exact test were used for comparison between groups. The continuous variables were expressed by mean ± standard deviation (SD), and independent-sample *t* test or rank sum test was used for comparison between groups. The variables with *P* value <0.1 were further involved in multivariate analysis. The Kaplan–Meier method was used to build the survival curves, and Cox regression was used for multivariate analysis. The test levels for entry and elimination of variables were, respectively, set at 0.05 and 0.10. The accuracy of the prediction model was evaluated by area under ROC curve (AUC). Based on the results of multivariate analysis, a nomogram was established. The C-index was used to verify the nomogram, and the test level *α* = 0.05. The verification group's data were put into the established prediction model to calculate the prediction results. The area under ROC curve was used to evaluate the differentiation degree of the model, and Hosmer–Lemeshow goodness-of-fit was used to test the calibration of the evaluation model. Ninety-five percent confidence intervals (95% CI) of hazard ratio (HR) were used as common measures to assess relative risk. All statistical analysis were performed using SPSS statistics 19.0 and R program (version 3.6.2). *P* < 0.05 were considered statistically significant.

## 4. Results

### 4.1. Demographic and Clinical Characteristics of the Model Group

The demographic and clinical characteristics of all subjects are presented in Table 1. The average age of all patients was (74.09 ± 9.00) years, including 772 patients aged 60–69 years (38.93%), 583 patients aged 70–79 years (29.40%), 597 patients aged 80–89 years (30.11%), and 31 patients over 90 years (1.56%). There were 1293 male patients (65.20%) with an average age of (74.30 ± 9.23) years and 690 female patients (34.80%) with an average age of (73.69 ± 8.53) years. The follow-up period was 12 months. 124 patients with VA (6.25%) were reported, and the average occurrence time was (7.9 ± 4.4) months. VA events included 14 cases of ventricular fibrillation, 1 case of pleomorphic ventricular tachycardia, 1 case of frequent ventricular tachycardia implanted with ICD, and other 108 cases of monomorphic ventricular tachycardia.

In terms of baseline data, the proportions of males, smoking, drinking, diabetes, and hyperlipidemia (HLP) in the VA group were higher than those in the non-VA group. In terms of ECG indexes, QTcd and Tp-e/QT in the VA group were higher than those in the non-VA group, and the SDNN index in HRV was lower than that in the non-VA group. In terms of biomarker indexes, NT-proBNP, Myo, cTnT, CK-MB, and CRP in VA group were higher than those in the non-VA group, while Ca^2+^ concentration in VA group was lower than that in the non-VA group. In terms of echocardiology, there were significant differences in left ventricular ejection fraction (LVEF), left ventricular end-diastolic diameter (LVEDD), left ventricular end-systolic diameter (LVESD), left atrial anterior-posterior diameter, left atrial superior-inferior diameter, left atrial left-right atrial diameter, and right atrial diameter (RAD) between the two groups. LVEF in the VA group was lower than that in the non-VA group, while the other indexes in the VA group were higher than those in the non-VA group.

### 4.2. Screening of Independent Predictors of VA

The risk factors affecting VA were screened by univariate analysis, and the variables with *P* value less than 0.1 were further involved in multivariate analysis. All the factors were analyzed by collinearity test, and the factors with collinearity did not enter into the multifactor analysis. Among the factors, age, Tp-e/QT, and NT-proBNP entered the multivariate analysis in the form of quartile. cTnT was more specific and sensitive than Myo and CK-MB in the diagnosis of myocardial injury in patients with acute myocardial infarction and heart failure [18], so cTnT was selected for multivariate analysis. Left atrial volume (LAV) was calculated by the combination of left atrial anterior-posterior diameter, left atrial superior-inferior diameter, and left-right atrial diameter (LAV ml = 4/3 *π* ∗ (left atrial anterior − posterior diameter mm/2) ∗ (left atrial superior-inferior diameter mm/2) ∗ (left atrial left-right diameter mm/2)/1000). The assignment of classification variables is described in Table 2, and the first level of the variable was defined as the base of comparison. Finally, gender, age (quartile), smoking, drinking, diabetes, HLP, QTcd, Tp-e/QT (quartile), SDNN, NT-proBNP (quartile), cTnT, Ca^2+^, LVEF, and LAV were selected for the Cox regression model. A forward stepwise regression method was used. The results showed that gender, age, HLP, QTcd, Tp-e/QT, LVEF, and LAV were independently correlated with the occurrence of VA. Age and Tp-e/QT  were dumb variables with the first quartile as the baseline (*P* < 0.05). The cumulative survival rate of all patients at the 12th month was between 93% and 94% (Figure 1). The time-dependent ROC curve of the model was drawn, and the AUC was 0.721 (95% CI: 0.669∼0.772) (Table 3 and Figures 2 and 3).

### 4.3. Comparison of Four Cox Regression Models including Different Factors

We selected different combinations of factors to establish Cox regression models for VA. The AUC of each model was compared, and the results are shown in Table 4 and Figure 4. The model's risk prediction probability was increased by 2.12% after adding ECG indexes to the prediction model, which included clinical baseline data, biomarker indexes and echocardiology indexes. The model's risk prediction probability was increased by 28.75% after adding the echocardiology indexes, which included clinical baseline data, ECG indexes, and biomarker indexes. The model's risk prediction probability was increased by 1.26% after adding the biomarker indexes, which included clinical baseline data, ECG indexes, and echocardiology indexes. Therefore, the Cox regression model with all types of factors had the highest prediction probability, in which echocardiology indexes had the greatest influence on the prediction efficiency, followed by ECG indexes (Table 4 and Figure 4).

### 4.4. Establishment of Nomogram

To simplify the complex model formula, we established a nomogram based on seven independent variables selected by the Cox regression model which included gender, age, HLP, QTcd, Tp-e/QT, LVEF, and LAV. Each factor had a score, and the total scores could be calculated (1.4–9.4) with the corresponding risk probability range 1-0. The C-index of the nomogram for predicting the overall risk of non-VA in 1 year was 0.785, suggesting that the nomogram had a good predictive value for the event (Figure 5).

### 4.5. Cox Regression Model Verification

Among 406 patients of the verification group, there were 40 patients with ventricular arrhythmias (9.85%). No significant difference was observed in gender, age, HLP, QTcd, Tp-e/QT, LVEF, and LAV between the model group and verification group (Table 5). Data of the verification group were substituted into the established Cox regression model, and the corresponding risk prediction probability value of each patient was calculated using the following equation:

(1) p^=1−S0texp∑i=1pβiXi−∑i=1pβiX¯i.

According to the risk prediction probability value, the ROC curve of the verification group was drawn, with AUC 0.73 (95% CI: 0.648∼0.818), indicating that the model had a certain distinguishing ability (Figure 6).

Calibration of the prediction model was evaluated by Hosmer–Lemeshow goodness-of-fit test. The prediction probability was sorted from small to large and divided into 10 groups according to ten points. The actual occurrence number and model prediction number of each group were calculated, respectively, and the actual incidence rate and predicted incidence rate were also calculated (Table 6). The actual incidence rate was expressed in the form of a bar chart, and the predicted incidence rate was expressed in the form of a curve (Figure 7). The results suggested that there was no statistical difference between predicted incidence rate and actual incidence rate (Hosmer-Lemeshow *χ*^2^ = 13.541, *P*=0.095). The predictive model had a good calibration.

## 5. Discussion

Despite the progress in risk prediction of VA [19], there has been no generally accepted large-sample-calculated model for predicting the occurrence of VA in elderly patients with CHD so far. Golukhova et al. [10] assessed the prognostic association of numerous biomarkers associated with future development of malignant ventricular arrhythmia (MVA) in patients with coronary artery disease (CAD) in a prospective, single-center observational cohort evaluation including 108 patients. They reported that prior MVA or syncope (OR: 11.1; 95% CI: 2.8–44.4; *P* < 0.01), abnormal heart rate turbulence (HRT) (ОR:13.6; 95% CI: 2.8–66.1; *P* < 0.01), and elevated plasma BNP (ОR:14.3; 95% CI: 3.2–65.0; *P* < 0.01) were independent MVA predictors. However, they did not discuss the predictive efficiency of the model. Compared with their study, larger-sized samples were enrolled and prospective model verification was performed in our study. Besides, we also compared the effects of different types of noninvasive indexes on the prediction performance of the model.

In this study, we established a multiparameter model for predicting VA in elderly patients with CHD and further verified its efficiency. Seven independent predictors, in order of importance of the relationship with outcome events, LVEF, LAV, HLP, QTcd, sex, Tp-e/QT, and age, were selected. Increased HLP, Tp-e/QT, QTcd, age, and LAV were risk factors (RR > 1), while female and increased LVEF were protective factors (RR < 1). This model can well predict the occurrence of VA in elderly patients with CHD (for model group, AUC: 0.721, 95% CI: 0.669∼0.772; for verification group, AUC: 0.73, 95% CI: 0.648∼0.818; Hosmer-Lemeshow *χ*^2^ = 13.541, *P*=0.095). In addition, we compared the prediction performance of different parameters. After adjusting the predictors, it was found that the combination of clinical indexes and ECG indexes could predict VA more efficiently than using clinical indexes alone.

VA is related to ventricular dysfunction and the extent of coronary disease. Among the echocardiography indexes, LVEF can accurately evaluate the ventricular function of patients with heart failure caused by various causes, and it is an independent and classical predictor of ventricular arrhythmia in patients with heart failure. It is generally believed that the changes of mechanical, morphological, electrophysiological characteristics, and neurohumoral remodeling of the heart during heart failure will not only aggravate ventricular hemodynamic disorders but also induce ventricular arrhythmias [20]. In an earlier study, Tracy et al. found that high-grade ventricular arrhythmia was associated with decreased rest and exercise LVEF, and the best predictor of ventricular arrhythmia was the decreased LVEF at rest, which worsened with exercise [21]. A number of researches had demonstrated that lower LVEF was an independent predictor of ventricular arrhythmia recurrence in CHD with secondary prevention ICD recipients [22–24]. LVEF is recognized as the gold standard of risk stratification for the occurrence of life-threatening ventricular arrhythmia. In this study, the echocardiography index LAV also entered the model. Increased LAV has been shown to be an independent risk factor for heart failure, stroke, and death. Previous studies have confirmed that enlarged LAV and impaired left atrial emptying fraction can predict the progression of heart failure and mortality [25, 26]. The hemodynamics of the left atrium and left ventricle influence and interact with each other [27]. In a retrospective study [28], Kaplan et al. found that the maximum LAV was associated with ventricular arrhythmias in patients after ICD implantation. In another study [29], Koilpillai et al. confirmed that left atrial width is related to the frequency of nonpersistent ventricular tachycardia. Similarly, in the present study, LVEF and LAV had been shown to be independent predictors of ventricular arrhythmias in elderly patients with CHD, and the prediction performance was improved by 28.75% after adding these two factors.

The ECG markers related to ventricular arrhythmias can reflect myocardial electrical instability, including Tp-e, Tp-e/QT, QTc, HRV, etc. The above-mentioned ECG markers reflect the heterogeneity of myocardial repolarization and plant nerve dysfunction. In recent years, studies have shown that Tp-e/QT can evaluate the time ratio of repolarization dispersion to the total duration of repolarization and can eliminate the confounding factors caused by heart rate variability and individual differences in QT intervals. So, Tp-e/QT is superior to Tp-e intervals and QT intervals and is becoming a more sensitive index for predicting ventricular arrhythmias [30–32]. In order to explore the predictability of the combination of multiple ECG parameters for ventricular arrhythmias, we added Tp-e/QT, QTcd, and HRV indicators for modeling and analysis, and it was confirmed that Tp-e/QT and QTcd could be used as independent predictors of ventricular arrhythmias in the elderly patients with CHD. In our study, the addition of ECG parameters increased the risk prediction probability of the model by 2.12%.

We also tried to identify the biomarkers to distinguish future ventricular arrhythmia risk. After univariate analysis, NT-proBNP and cTnT entered the multivariate analysis, but neither of them became independent predictors of VA. However, it cannot be denied that there is a correlation between NT-proBNP & cTnT and ventricular arrhythmias in patients with coronary heart disease. BNP and NT-proBNP have been proved to be equivalent and sensitive markers of systolic and diastolic function during left ventricular injury and can help identify high-risk groups of adverse cardiovascular events [33]. Lindholm et al. [34] confirmed that NT-proBNP and hs-cTnT had greater prognostic value than any other biomarkers for cardiovascular outcomes. In a study of ventricular arrhythmias in children, Mazurek et al. [35] found that the level of NT-proBNP increased with the severity of the ventricular arrhythmia, and the determination of NT-proBNP is helpful for the diagnosis and grading of ventricular arrhythmias.

This model is helpful for clinicians to understand important risk factors affecting VA occurrence in elderly patients with CHD so as to reduce the incidence of VA and improve the survival rate of patients. In addition, the seven indexes in the model are economical, noninvasive, and convenient and easy to obtain, with the manipulation unlimited by hospital conditions.

## 6. Study Limitation

Drug use had not been analyzed. The RR values of some of the seven factors in the model were close to 1, so we could not rule out the influence of drugs on the outcome and other unknown confounding factors, which could result in bias and affection on the result. In the retrospective case collection, the collection of NT-proBNP and cTnT in some cases lagged behind the event occurrence, which failed to reflect the real concentration at the event time, thus affecting the accuracy. Besides, this study was a single-center cohort evaluation, so multicenter and larger sample studies are still needed to optimize and verify the model in the future.

## 7. Conclusions

LVEF, LAV, QTcd, Tp-e/QT, gender, age, and HLP were independent predictors of VA risk in elderly patients with CHD. Among these factors, the echocardiology indexes LVEF and LAV had the greatest influence on the predictive efficiency of the model, followed by ECG indexes, QTcd and Tp-e/QT. After verification, the model had a good degree of differentiation and calibration, which can provide a certain reference for clinical prediction of the VA occurrence in elderly patients with CHD.

## Figures and Tables

**Figure 1:** The cumulative survival rate of all patients in 12 months.

**Figure 2:** Cumulative survival function curves of each classified variable (a)–(g). Indexes are grouped by median (d, f, g). (a) Cumulative survival function curve of gender. (b) Cumulative survival function curve of age. (c) Cumulative survival function curve of HLP. (d) Cumulative survival function curve of QTcd. (e) Cumulative survival function curve of Tp-e/QT. (f) Cumulative survival function curve of LVEF. (g) Cumulative survival function curve of LAV.

**Figure 3:** ROC curve of the model group.

**Figure 4:** AUC comparisons of each model.

**Figure 5:** Nomogram for predicting the overall risk of non-VA in 1 year.

**Figure 6:** ROC curve of verification group.

**Figure 7:** Distribution map of actual incidence rate and predicted incidence rate.

**Table 1:** Comparison of demographic and clinical characteristics between VA and non-VA groups.

Characteristic	VA (*N* = 124)	Non-VA (*N* = 1859)	*z*/*χ*^2^	*P* value
Male, *n* (%)	103 (83.06%)^*∗∗*^	1190 (64.01%)	18.597	*P* ≤ 0.001
Age, mean (SD), y	75.44 (8.70)	74.00 (9.01)	−1.770	0.077
Height, mean (SD), cm	167.61 (6.64)^*∗∗*^	165.08 (7.69)	−3.708	*P* ≤ 0.001
Weight, mean (SD), kg	69.33 (12.29)	68.00 (11.19)	−1.807	0.071
BMI, mean (SD), kg/m^2^	24.60 (3.80)	24.87 (3.45)	−0.438	0.662
Smoking, *n* (%)	48 (38.7%)^*∗*^	570 (30.66%)	3.510	0.040
Drinking, *n* (%)	31 (25%)^*∗*^	334 (17.97%)	3.829	0.036
Diabetes, *n* (%)	60 (48.39%)^*∗∗*^	673 (36.20%)	7.407	0.005
Hypertension, *n* (%)	88 (70.97%)	1346 (72.40%)	0.120	0.399
HLP, *n* (%)	94 (75.81%)^*∗∗*^	1083 (58.26%)	14.840	*P* ≤ 0.001
Atherosclerosis, *n* (%)	14 (11.29%)	222 (11.94%)	0.047	0.483
QTcd, mean (SD), ms	37.77 (27.61)^*∗∗*^	27.27 (18.47)	−4.313	*P* ≤ 0.001
Tp-e/QT, mean (SD)	0.23 (0.04)^*∗∗*^	0.21 (0.04)	−3.858	*P* ≤ 0.001
SDNN, mean (SD), ms	91.99 (32.35)^*∗∗*^	103.90 (38.36)	−3.744	*P* ≤ 0.001
SDANN, mean (SD), ms	98.06 (48.02)	102.36 (50.91)	−1.529	0.126
RMSSD, mean (SD), ms	43.26 (38.05)	38.83 (37.84)	−0.931	0.352
PNN50 (%), mean (SD)	4.69 (6.15)	4.76 (7.67)	−0.502	0.615
NT-proBNP, mean (SD), pg/ml	1730.94 (4704.69)^*∗∗*^	891.08 (3251.88)	−4.452	*P* ≤ 0.001
Myo, mean (SD), ng/ml	133.57 (336.15)^*∗*^	46.94 (101.67)	−2.445	0.014
cTnT, mean (SD), ng/ml	0.35 (0.97)^*∗∗*^	0.22 (1.69)	−6.343	*P* ≤ 0.001
CK-MB, mean (SD), ng/ml	10.88 (18.58)^*∗∗*^	8.23 (23.66)	−4.058	*P* ≤ 0.001
CRP, mean (SD), mg/dl	0.90 (2.45)^*∗*^	0.61 (1.81)	−2.403	0.016
K^+^, mean (SD), mmol/L	3.88 (0.40)	3.90 (0.42)	−0.551	0.582
Ca^2+^, mean (SD), mmol/L	2.20 (0.10)^*∗∗*^	2.24 (0.13)	−3.173	0.002
LVEF, mean (SD), %	49.50 (11.63)^*∗∗*^	58.95 (7.66)	−9.334	*P* ≤ 0.001
Interventricular septal thickness, mean (SD), mm	10.71 (1.37)	10.93 (1.37)	−1.218	0.223
LVPW, mean (SD), mm	10.08 (0.96)	10.11 (1.05)	−0.027	0.979
LVEDD, mean (SD), mm	48.40 (6.10)^*∗∗*^	45.36 (4.89)	−5.640	*P* ≤ 0.001
LVESD, mean (SD), mm	35.55 (7.11)^*∗∗*^	31.07 (4.91)	−7.373	*P* ≤ 0.001
Left atrial anterior and posterior diameter, mean (SD), mm	36.75 (5.21)^*∗∗*^	35.33 (4.51)	−3.087	0.001
Left atrial superior and inferior diameter, mean (SD), mm	55.06 (5.53)^*∗∗*^	51.47 (5.69)	−6.484	*P* ≤ 0.001
Left atrial left and right atrial diameter, mean (SD), mm	38.54 (4.26)^*∗∗*^	36.18 (4.42	−5.744	*P* ≤ 0.001
E-peak, mean (SD), m/s	0.68 (0.20)	0.69 (0.21)	−0.208	0.835
A-peak, mean (SD), m/s	0.90 (0.26)	0.90 (0.23)	−1.897	0.058
Inner diameter of ascending aorta, mean (SD), mm	31.46 (3.79)	32.13 (3.57)	−1.560	0.119
Stroke volume, mean (SD), ml	52.17 (14.49)	55.30 (13.29)	−1.863	0.063
Internal diameter of right atrium, mean (SD), mm	35.50 (4.98)^*∗∗*^	32.77 (4.25)	−5.507	*P* ≤ 0.001

LVPW: left ventricular posterior wall; ^*∗*^means comparison between the two groups *P* < 0.05, ^*∗∗*^means comparison between the two groups *P* < 0.01.

**Table 2:** Variable assignment description.

Variable name	Variable type	Classified variable coding
Gender	2 classification	Male = 0, Female = 1
Age, year (quartile)	Ordered grade	60∼66 year = 1
		67∼75 year = 2
		76∼82 year = 3
		Above 82 year = 4
Smoking	2 classification	Nonsomker = 0, smoker = 1
Drinking	2 classification	Nondrinker = 0, drinker = 1
Diabetes	2 classification	Nondiabetes = 0, diabetes = 1
HLP	2 classification	Non-HLP = 0, HLP = 1
QTcd (ms)	Continuous variable	
Tp-e/QT (quartile)	Ordered grade	0∼0.192 = 1
		0.1921∼0.224 = 2
		0.2241∼0.245 = 3
		Above 0.245 = 4
SDNN	Continuous variable	
NT-proBNP, pg/ml (quartile)	Ordered grade	0∼63.01 = 1
		63.02∼171.4 = 2
		171.41∼474.1 = 3
		Above 474.1 = 4
cTnT (ng/ml)	Continuous variable	
Ca^2+^ (mmol/L)	Continuous variable	
LVEF (%)	Continuous variable	
LAV (ml)	Continuous variable	

**Table 3:** Multivariate analysis of model group by Cox regression.

Variable code	Variable	*B*	SE	Wald	*P* value	HR (95% CI)
*X*_1_	Sex	−0.913	0.246	13.830	*P* ≤ 0.001	0.401 (0.248–0.649)
*X*_2_^*∗∗*^	Age (2)	0.647	0.270	5.744	0.017	1.910 (1.125–3.241)
*X*_2_^*∗∗∗*^	Age (3)	0.009	0.301	0.001	0.975	1.009 (0.560–1.820)
*X*_2_^*∗∗∗∗*^	Age (4)	0.672	0.279	5.808	0.016	1.959 (1.134–3.384)
*X*_3_	HLP	1.832	0.234	61.474	*P* ≤ 0.001	6.245 (3.951–9.872)
*X*_4_	QTcd	0.011	0.004	8.940	0.003	1.011 (1.004–1.018)
*X*_5_^*∗∗*^	Tp-e/QT (2)	0.465	0.308	2.283	0.131	1.592 (0.871–2.910)
*X*_5_^*∗∗∗*^	Tp-e/QT (3)	0.687	0.303	5.136	0.023	1.988 (1.097–3.601)
*X*_5_^*∗∗∗∗*^	Tp-e/QT (4)	0.890	0.303	8.644	0.003	2.435 (1.345–4.408)
*X*_6_	LVEF	−0.121	0.009	165.20	*P* ≤ 0.001	0.886 (0.870–0.902)
*X*_7_	LAV	0.016	0.007	5.268	0.022	1.016 (1.002–1.030)

**Table 4:** Comparison of AUC of each model.

Test variables	AUC (95% CI)	Standard error	*P* value
All types of factors	0.721 (0.669–0.772)	0.026	*P* ≤ 0.001
Factors except ECG indexes	0.706 (0.652–0.761)	0.028	*P* ≤ 0.001
Factors except echocardiology indexes	0.560 (0.504–0.616)	0.029	0.025
Factors except biomarker indexes	0.712 (0.659–0.756)	0.027	*P* ≤ 0.001

**Table 5:** Comparison of risk factors between model group and verification group.

	Model group (*N* = 1983)	Verification group (*N* = 406)	*P* value
Gender (male)	1293 (65.20%)	270 (66.50%)	0.668
Age			0.374
60∼66 years	544 (27.43%)	120 (29.56%)	
67∼75 years	506 (25.52%)	99 (24.38%)	
76∼82 years	502 (25.32%)	66 (16.26%)	
Above 82 years	431 (21.73%)	121 (29.8%)	
HLP	1177 (59.35%)	225 (55.42%)	0.145
QTcd (ms)	27.92 ± 19.33	28.40 ± 20.41	0.885
Tp-e/QT			0.266
0∼0.19	500 (25.21%)	63 (15.52%)	
0.20∼0.22	510 (25.72%)	92 (22.66%)	
0.23∼0.24	506 (25.52%)	121 (29.8%)	
Above 0.24	467 (23.55%)	130 (32.02%)	
LVEF (%)	58.24 ± 8.38	58.58 ± 8.38	
LAV (ml)	35.59 ± 11.34	34.67 ± 10.43	0.259

**Table 6:** Actual incidence rate and predicted incidence rate.

Tenth quantile	Predicted incidence rate (%)	Actual incidence rate (%)
1	0.44	0
2	0.75	2.01
3	1.02	0
4	1.34	2.53
5	1.71	0
6	2.11	2.01
7	2.60	3.03
8	3.31	4.04
9	4.75	5.56
10	44.8	43.65

## Data Availability

The data used to support the findings of this study are available from the corresponding author upon request.
